The article "The Effects of Rural Residents' Sleep Quality on the Incidence of Agricultural Injuries: A Meta-Analysis" was retracted in 2023. Reasons: signs of a paper mill; suspected computer-generated content; unreliable results or conclusions; concerns about the data.

# The Effects of Rural Residents' Sleep Quality on the Incidence of Agricultural Injuries: A Meta-Analysis

**DOI:** 10.1155/2022/3832535

**Published:** 2022-07-13

**Authors:** Xiaobing Zhai, Li Cao, Bing Zhang, Qiao Li

**Affiliations:** ^1^Department of Biostatistics, International School of Public Health and One Health, Hainan Medical University, Haikou 571199, China; ^2^Department of Mathematical Statistics, International School of Public Health and One Health, Hainan Medical University, Haikou 571199, China

## Abstract

To collect relevant literature on the impact of rural residents' sleep quality on the incidence of agricultural injuries, the search time range is 1990～2019. We use RevMan 5.3 software for statistical processing. A total of 7 articles were included. Meta-analysis showed that sleep quality was closely related to agricultural injury. The combined effect was 1.49, 95%*CI* [1.31, 1.70], *Z* = 5.93, *P* < 0.00001. The difference was statistically significant, so poor sleepers had a higher incidence of agricultural injuries than good sleepers. Sleep disturbances and agricultural injuries are two common and significant health problems. Investigations suggest that sleep might increase the risk of agricultural injuries. The aim of the present study was to systematically review and meta-analyze the predictive effect of sleep on agricultural injuries.

## 1. Introduction

Agricultural injury is a significant public health problem globally [1]. Since the 1990s, injuries to agricultural workers have been studied extensively, particularly in the developed countries, and high rates of mortality and morbidity have been reported.

The fatality rate for agriculture was eight times higher compared to all industries combined [2]. As we all know, agriculture is a major occupation in the world and is closely related to many health problems. Agriculture is the industry with the highest incidence of occupational injuries in the UK, ranking fourth among the most vulnerable industries in the US, and it is also one of the most dangerous occupations in Canada [3, 4]. In 2019, the incidence of fatal injuries was 23.1 injuries per 100,000 full-time equivalent (FTE) workers in agriculture compared to 3.5 per 100,000 in all other industries combined [5]. The rate of non-fatal injuries was 5.2 injuries per 100 FTE workers in agriculture and 2.8 per 100 in all other industries combined [6]. The high rates represent a hard pressing problem of unintentional occupational injury in modern agriculture.

Previous studies have shown that the injury rate is higher for people engaged in agriculture than those in other occupations, and those in rural areas are higher than those in urban areas [2, 7]. Therefore, ensuring adequate sleep duration for farmers is of great importance [8]. In recent years, the effect of sleep quality on the incidence of agricultural injuries has received much attention.

Although some studies have clarified the relationship between agricultural damage and sleep quality, little research has been done on the potentially important and correctable relationship between sleep quality and agricultural damage injury [9].

So, agricultural damage and the relationship between sleep quality and the effect of sleep quality on the incidence of agricultural injury are still in a narrow surface understanding; in order to further clarify the effect of sleep quality on the incidence of agricultural injury and provide reference for third-level prevention, this article made a meta-analysis of the effect of sleep quality on the incidence of agricultural injuries. The purpose of this study is to retrieve relevant research on the effect of sleep quality on agricultural injuries at home and abroad and to provide new methods and ideas for the study of the effect of sleep quality on the incidence of agricultural injuries.

## 2. Materials and Methods

### 2.1. Literature Search

Chinese search terms were “sleep quality” or “agricultural injury” or “rural residents” or “sleep disorder” or “agricultural injury” or “rural residents.” English search terms were “sleep quality” or “agricultural injuries” or “Country dweller” or “sleep quality” or “farm injuries” or “Country dweller.” Different database retrieval methods are different. In the retrieval process, in order to ensure that all the studies related to research are retrieved and to improve the reliability and practicality of the research, different retrieval formulas should be formulated in the retrieval process in combination with the retrieval characteristics of the database.

### 2.2. Literature Inclusion and Exclusion Criteria

Inclusion criteria were as follows: ①relevant research on the effects of rural residents' sleep quality on agricultural injuries published between 1990 and 2019; ② the sample size in the literature is clearly described; ③ research or literature has specific publication period; and ④ the full text can be retrieved in the database.

Exclusion criteria were as follows: ① repetitive publication of various studies; ② there are obvious defects in the research design; ③ poor literature quality; and ④ poor data integrity.

### 2.3. Sleep Quality

The study reported a clear sleep time. The sleep duration was calculated based on reported sleep and awakening times, and the responses were (1) high sleep quality >7 hours and (2) poor sleep quality ≤7 hours.

### 2.4. Literature Screening and Data Extraction

Two team members read the abstract and full text of the articles and extracted data from articles. If the opinions are not uniform, a third person is required to discuss until the opinions are agreed. According to the inclusion and exclusion criteria, the screened articles will be screened first, and the initially included articles will be screened again by reading the full text [10].

### 2.5. Literature Quality Evaluation

At present, countries around the world have not formulated specific uniform standards for current research. This study is based on *the Strengthening the Reporting of Observational Studies Epidemiology* (STROBE). The following is an assessment of the various aspects of the cross-sectional study: (1) stochastic method; (2) withdrawal or loss of access; (3) whether it clearly states the effective response rate and the effective response rate>90%; (4) whether quality control is performed; (5) whether the statistical method is reasonable, etc. (6) According to the above standards, the studies is divided into three categories: low risk, uncertain, and high risk, as shown in Table 1.

Literature quality score (up to 6 points): 0–2 points are low quality and 3 points and above are high quality [11]. In order to ensure a correct and reasonable quality assessment of each literature and improve the reliability of the study, two team members read the abstract and full text of the articles and extracted data from articles; if the opinions are not uniform, a third person is required to enter into discussion until the opinions are agreed.

### 2.6. Statistical Analysis

Meta-analysis was conducted using RevMan 5.3 software; RevMan 5.3 official version is a meta-analysis tool with quite practical functions. RevMan 5.3 official version has the characteristics of simple operation and intuitive results. It is one of the more mature special meta-analysis software applications at present. At present, it can mainly complete the systematic evaluation of intervention research and diagnostic test research, as well as the systematic evaluation of the other two higher perspectives.

#### 2.6.1. Summary Analysis and Heterogeneity Test of the Effects of Rural Residents' Sleep Quality on the Incidence of Agricultural Injuries

We use RevMan 5.3 Meta to summarize and merge the data of the articles and draw the forest map. When *I*^2^ <50%, it indicates that the heterogeneity between the studies is small and can be ignored; then, the fixed-effect model is selected. When *I*^2^ ≥50%, it indicates that there is substantial heterogeneity. Under the premise of ensuring homogeneity, the statistical analysis of data is carried out using a random effect model. When there is no heterogeneity between studies, the analysis results of two models have good consistency, and the difference is not statistically significant. When there is no heterogeneity between studies, the confidence interval calculated by the selected fixed-effect model is small, and the results are more open.

#### 2.6.2. Publication Bias

The study used a funnel plot to estimate the existence of publication bias. The abscissa and ordinate in the funnel chart are sleep quality and sample size, respectively. If the funnel chart is roughly symmetrical, it means that there is no obvious publication bias in the articles included in the institute; if the funnel chart is skewed, it means that the study has publication bias. Although the funnel chart is relatively intuitive and simple, it is easily affected by the observer's subjective consciousness, so sometimes the most accurate test cannot be made [11].

## 3. Results

### 3.1. Literature Search

After the search terms are determined, when searching, in order to improve the reliability and practicality of research, different search formulas should be formulated in accordance with the search characteristics of the database to ensure that all the articles related to the research are retrieved. The file retrieval steps are shown in Figure 1.

### 3.2. Study Characteristics and Quality Evaluation

Table 2indicates that among the 7 included articles [12–18],

1. There are 3 studies that clarify the random method and type of study, 1 study only mentions the random method, 2 studies only mention the type of study, and 1 study is not clear about its random method and type.
2. There are 7 articles of high-quality research included. Among them, there are 2 articles with a score of 5, 3 articles with a score of 4, and 2 articles with a score of 3.
3. The included studies are generally large-sample current studies. Among them, there are 3 large-sample studies (with a sample size of at least 2000); 2 medium-sized studies (with a sample size of at least 1000); and 2 small-sample studies (sample size within 1000).

### 3.3. A Summary Analysis of the Effects of Rural Residents' Sleep Quality on the Incidence of Agricultural Injuries

In related studies, the heterogeneity test results showed that there was no statistical heterogeneity between them (*I*^2^ <50.0%, *P* > 0.05), so the fixed-effect model was used for the merger analysis. As shown in Figure 2, there were 2548 people with low sleep quality, 397 people injured by agriculture, accounting for 15.46%, 12815 people with high sleep quality, and 1457 people injured by agriculture, accounting for 11.37%. The combined effect size was 1.49, 95%*CI* [1.31, 1.70], *Z* = 5.93, *P* < 0.00001, indicating that there was a statistically significant difference in the incidence of agricultural injuries between people with low sleep quality and those with high sleep quality.

### 3.4. Publication Bias and Sensitivity Analysis

This study uses a funnel chart to evaluate the publication bias of the included articles. According to Figure 3, the funnel chart is basically symmetrical, indicating that there is no obvious publication bias in the articles. In order to conduct sensitivity analysis and compare the changes in the total effect size of each study, the difference of the effect sizes obtained from different combined models is compared. Meta-analysis results show that there is no essential difference in the merged results, indicating that the research results are relatively stable [17].

## 4. Discussion

The current meta-analysis showed that sleep could significantly affect agricultural injury. In particular, poor sleep quality had a higher risk of agricultural injury compared to higher sleep quality.

Previous studies showed that sleep quality has been associated with a wide range of health outcomes, including cognitive[19], psychosocial [1], and cardiometabolic health [2], as well as specific conditions such as type 2 diabetes [3], cardiovascular disease [4], stroke [5], and obesity [6]. Sleep is recognized as a central concern for population health and is one of the three pillars of a healthy lifestyle, including diet, exercise, and sleep. Sleep is an important means to relieve fatigue, restore physical strength, and promote health. Sleep quality is closely related to human physiology and psychology and plays an important role in maintaining human health, work efficiency, and quality of life [7]. The included studies [12–14] showed that under the control of variables other than sleep, the incidence of agricultural industrial injuries in people with low sleep quality was higher than that in people with high sleep quality, and shortened sleep time and poor sleep quality could significantly increase the risk of agricultural industrial injuries. Therefore, when assessing the occupational safety of farmers, while considering other factors, sleep duration and sleep quality should also be considered.

This phenomenon has to attract extensive social attention. Adequate sleeping is required for farmers to maintain alertness to remain productive on the job. The study [15] indicated that sleep quality and work-related injuries are generally applicable to a wider agricultural population. Limited sleep time due to seasonal is highly correlated with the risk of injuries to farmers; when evaluating the relationship between agricultural injury and sleep quality, it is necessary to consider the effects of seasonal changes in sleep on agricultural injury; these comparison results further indicate the relationship between sleep quality and work-related injuries. As we all know, poor sleep quality will affect the mental state the next day, including drowsiness, inattention, memory, decision making, and other problems. Poor mental state was significantly correlated with agricultural injury. These also support the results of our study.

All in all, sleep quality is significantly associated with agricultural injuries. Those with poor sleep quality reported higher agricultural injuries than those with good sleep quality. Although there are some articles on the relationship between agricultural injuries and sleep quality, there is little research on the potentially important and correctable relationship between sleep behavior and injuries. The relationship with sleep quality and the effects of agricultural injuries on sleep quality are still in a narrow superficial understanding [8, 28].

## 5. Limitations of Research

1. Because there are not many high-quality domestic and foreign articles on the effects of rural residents' sleep quality on the incidence of agricultural injuries.
2. Due to the influence of factors such as the study characteristics, research methods, random types, evaluation methods, social and living environment, and so on of the included research, the heterogeneity of the research results may increase, which may deviate from the direction and problems of the research. In the included articles, sleep quality is a subjective evaluation indicator, which is greatly affected by human and psychological factors, and other objective evaluation indicators and methods have not been adopted. Therefore, it may affect the authenticity and reliability of the research results.

## 6. Conclusions

Reduced sleep hours and quality may increase the risk of agricultural work-related injuries in farmers. Findings of this study underscore an important occupational safety issue facing millions of farmers in world and verify the association between lack of sleep and risk of agricultural injuries [29–32].

## Figures and Tables

**Figure 1:** Content indexing steps.

**Figure 2:** Forest map of the impact of rural residents' sleep quality on the incidence of agricultural injuries.

**Figure 3:** Funnel chart of the effects of rural residents' sleep quality on the incidence of agricultural injuries.

**Table 1:** Literature quality evaluation.

Grading	Description	Score
Stochastic method	Identify random methods and types	2
	Only mentions the random method but does not specify its type	1
	The random method is inappropriate or only mentions its type or is unclear	0

Withdrawal or loss of access	Yes	0
	No	1

Whether it clearly states the effective response rate and the effective response rate> 90%	Yes	1
	No	0

Whether quality control is performed	Yes	1
	No	0

Whether the statistical method is reasonable	Yes	1
	No	0

**Table 2:** Study characteristics.

Number	Inclusion study	Stochastic method	Sample size	Withdrawal or loss of access	Effective response rate	Score
[12]	Huiping Zhu 2014	Multistage sampling	2264	Yes	Yes	3
[13]	Luo Fengqi 2016	Random cluster sampling	624	Yes	Yes	5
[14]	Zhao Na 2011	Group sampling	1921	No	No	5
[15]	Rebbecca Lilley 2012	Mention only types	4439	No	Yes	4
[16]	James A Dosman MD2013	Mention only types	5502	No	Yes	4
[17]	M. W. Postel2009	Not sure	1551	Yes	Yes	3
[18]	LorannStallones2006	Mention only random	262	No	No	4

## Data Availability

The experimental data used to support the findings of this study are available from the corresponding author upon request.
